# Construction of Urban Flood Disaster Emergency Management System Using Scenario Construction Technology

This article has been retracted.

**DOI:** 10.1155/2022/8048327

**Published:** 2022-03-15

**Authors:** Xianghai Li, Yixin Wang

**Affiliations:** ^1^School of Emergency Management, Henan Polytechnic University, Jiaozuo, Henan 454003, China; ^2^School of Civil Engineering, Henan Polytechnic University, Jiaozuo, Henan 454003, China

## Abstract

Due to the global climate anomaly, ecological environment damage, human activities, and other reasons, flood disaster has become a major threat to mankind. The emergency rescue resources under different subject management and different emergencies have different characteristics, attributes, and management modes, which restrict the unified dispatching, overall management, and efficient utilization of the comprehensive rescue command platform. The frequent occurrence of natural disasters can not only easily affect the public security of society but also pose a great threat to the safety of Chinese people's lives and property. As the first-line person in charge of China's response to natural disasters, local governments cannot deal with natural disasters well. More than thousands of people die from natural disasters in China every year. The economic losses caused amounted to hundreds of billions. The occurrence of various floods and natural disasters not only affects the local economic and social development but also relates to the production and life of the local people, and the stability of the local society and national unity. How to effectively deal with flood disaster is also an important index system to test the execution and management ability of the Party and the government. Therefore, it is necessary to deeply study flood disaster from the theoretical height, hoping to provide reference theoretical support and practical guidance for local county-level government flood disaster emergency management. At the beginning of the urban flood disaster, how to choose an appropriate response plan and implement it in time is an important way to effectively reduce disaster losses. Starting with the basic concept of flood disaster, this study studies and discusses the related theories of flood disaster emergency management, introduces the general situation of flood disaster emergency management, and analyzes the application of scenario construction technology in emergency management.

## 1. Introduction

As a kind of natural disasters, floods frequently occur and pose a great threat to the security and stability of human society for many years due to the combined effects of many factors (complex natural and geographical environment, excessive human activities, etc.). With the rapid development of society and economy, accidents in key industries and fields such as mining, transportation, construction, civil explosion, and dangerous chemicals occur from time to time, which poses great harm to the safety of life and property of cities and people [1]. Earthquakes, mountain torrents, tsunamis, and other natural disasters frequently occur, which bring people life and property losses [2]. Floods and floods not only threaten people's life safety to a certain extent, but also the economic and property losses caused by floods and floods will seriously hinder the development of local society and economy, even the process of social stability and modernization. Affected by the abnormal global climate, the coastal cities in southeast China have been repeatedly hit by major floods and floods, causing heavy casualties and property losses, which put forward higher requirements for the government's emergency management [3]. Despite the steady progress of urban emergency management and disposal, the government faces great pressure in dealing with emergencies due to the suddenness, diffusion, uncertainty, and variability of development and change [4]. Flood disaster caused the Yellow River to burst its banks, and the losses in the affected areas exceeded 100 million yuan, which had a great impact on people's production and life [5].

Natural disasters have caused enormous losses to China. Facing the destruction of natural disasters, China has also accumulated a lot of effective emergency management experience, promulgated laws and regulations on emergency management of natural disasters, issued emergency management plans for natural disasters, and established an emergency management system for natural disasters [6]. Strengthening disaster prevention and mitigation, reducing the losses caused by various disasters, plays an important role in building a harmonious society and promoting social stability and is an important foundation for ensuring the safety of people's lives and property and building a harmonious society [7]. In China, county-level governments are often in the front line of flood disaster emergency management, but their emergency management ability for flood disaster is restricted by the lack of many resources and personnel capacity [8]. After the disaster, if the appropriate emergency response plan is started in time within the “golden time” of emergency response, the further expansion of the impact of flood disaster can be effectively controlled [9]. It is an important and urgent task for city managers to effectively deal with all kinds of emergencies and build a comprehensive urban emergency platform, and it is also a key measure to adapt to the current situation [10].

To sum up, a fast and effective emergency plan generation method plays an important role in supporting government emergency decision-making and command and improving emergency work efficiency. Building a unified emergency resource structure model is a basic link in the construction of an emergency resource system, such as the construction of an emergency resource input guarantee mechanism and the improvement of emergency resource guarantee and mobilization mechanism [11]. It is conducive to improving the support capacity of emergency rescue, realizing the effective integration and optimal allocation of emergency resources under the background of the urban comprehensive emergency platform and oriented by emergency demand, and realizing the agile response under the state of emergency rescue [12]. Theoretically, it can enrich and improve the research content of the emergency plan generation method [13]. Through natural disaster emergency management, the economic losses caused by natural disasters are reduced, the safety of people's lives and property is ensured, and the good development of social and economic order is promoted [14]. On the one hand, the study of natural disasters is helpful to deal with the political problems in disaster prediction, disaster control, and disaster aftermath, and to the establishment and development of the new science of disaster politics. On the other hand, the research on flood disaster emergency management of county-level government is conducive to adapt to the development trend of globalization.

## 2. Related Work

Literature [15] holds that the decision support system for emergency management is composed of a database subsystem, plan database subsystem, case database subsystem, method database subsystem, and model database subsystem. Literature [16] puts forward the establishment of an emergency management model based on system control, including strategic capability, development capability, and process capability (including prevention, preparation, emergency response, and prevention). It holds that we should improve the strategic awareness of emergency management, advocate the development concept and strategy of internalization and institutionalization of risk awareness, improve the development capability of risk prevention, reduce the vulnerability of communities to disasters, improve the adaptability of communities to risks, and establish a comprehensive system combining crisis prevention and crisis response. Literature [17] puts forward that local government is the main body of public crisis management. According to the decentralization efficiency theory of government management and the type attribute of public crisis, local government is the natural subject of most public crisis management. Literature [18] puts forward the similarity measurement method of CBR, which can realize effective case representation and make its development prospect in the computer field broader. Literature [19] advocates that government authorities should organize formal official institutions to deal with various natural or man-made emergencies. Literature [20] puts forward the concept of representation ontology in ontology to describe and represent the characteristic attributes of historical cases and integrates historical cases into standardized expressions. Literature [21] expounds on the current construction of earthquake emergency basic database from the aspects of significance, database definition, basic data content, database function, database building methods and principles, etc. Literature [22] on the basis of matter element representation, by analyzing the conviction and sentencing system of criminal law, this study puts forward a general and effective four-level representation method of cases [23] Starting from the present situation of China's natural disaster emergency management, this study systematically analyzes the research progress in the field of a natural disaster emergency management and points out the problems in theory and practice of China's natural disaster emergency management. Literature [24] holds that the establishment of natural disaster emergency management system suitable for China's national conditions is the basis for improving China's natural disaster emergency management: the formulation and implementation of the emergency plan are the key measures to standardize disaster emergency management and improve disaster emergency rescue capability; fast and accurate acquisition and evaluation of disaster information are an effective guarantee for disaster emergency management; establishing practical emergency management system is the fundamental way to improve disaster emergency management level and work efficiency.

## 3. Connotation, Characteristics, and System Composition of Natural Disaster Emergency Management

### 3.1. Connotation of Natural Disaster Emergency Management

The concept of crisis management originated from enterprises, which refers to the management of crisis events by enterprises. With the increase in social requirements for the government's responsibility for crisis events, the concept of government crisis management came into being [25]. Among them, the disasters caused by heavy rainfall, melting of snow and ice, ice, dam break, storm surge, and other reasons, such as the increase in water volume in rivers, lakes, and coastal areas, the flood caused by rising water level and flash floods, are called flood disasters [26]. The disasters caused by heavy rain, heavy rain, or long-term rainfall are called waterlogging disasters, which result in a large amount of accumulated water and runoff and untimely drainage, resulting in waterlogging and flooding of land and houses. Emergency management of natural disasters belongs to the category of government emergency management. Therefore, the definition of emergency management of natural disasters cannot be divorced from government crisis management and talked about crisis management of natural disasters [27]. That is, the government and other public institutions, in the process of preprevention, incident response, in-process handling, and after-care recovery of emergencies, adopt a series of necessary measures and apply science, technology, planning and management, and other means to ensure people's lives, health, and property safety [28]. After the implementation of the emergency plan, whether the disaster situation is effectively controlled, whether the actual problems are solved, and whether the casualties, property losses, and environmental changes are effectively directly controlled determine the effectiveness and practicability of the emergency plan. Based on this, the content of urban flood disaster case representation is designed as shown in Figure 1.

Activities related to promoting harmonious social development are often collectively referred to as flood disasters because flood disasters and rain disasters often simultaneously or continuously occur in the same area, and sometimes it is difficult to accurately define them [29]. Due to the difficulty of obtaining information at the beginning of an emergency and the urgency of time, emergency decision-making faces various uncertainties. At present, there is no general mature and systematic method for emergency decision-making. The commonly used strategies mainly include the rapid decision analysis method, decision support model method, plan-based decision-making method, and case-aided decision-making method. The goal of the emergency rescue stage of urban emergencies is to reduce the damage of emergencies as much as possible through effective actions, including casualties, property losses, and environmental damage. The traditional emergency management pays more attention to the response after the crisis, ignores the influencing factors causing the outbreak of the crisis, looks for the root causes of the crisis through the manifestations of the crisis, analyzes the impact scope and losses caused by the crisis, and takes countermeasures to effectively reduce the risk of the crisis. Therefore, effective emergency management needs to reduce the impact scope caused by the crisis, find out the source of the crisis, pay attention to the influencing factors of the crisis, and then improve the management to reduce losses. Crisis management can be divided into six different stages: crisis prevention, crisis avoidance, crisis management preparation, crisis control, crisis resolution, and profit from the crisis. In order to solve many practical problems in the process of emergency decision-making, many scholars have studied related problems by using the fast decision analysis method or decision support model method and have obtained some research results. Some application examples have been adopted by the government in the actual decision-making process, which also constitutes a part of the current emergency decision-making of urban flood disaster. After a disaster, the government and various rescue units need to accurately and quickly match rescue measures according to the nature of the disaster. The task of emergency management is to control the situation as much as possible, control the losses within a certain range in crisis events, and try to regain control of government emergency management after things get out of control. It refers to a series of planned and organized management processes carried out by the government to deal with emergencies. It is the activities of the government and other public organizations to reduce government emergency management through measures such as detection, early warning, prevention, emergency handling, evaluation, and recovery under the guidance of scientific management concepts.

### 3.2. Composition of Natural Disaster Emergency Management System

In order to effectively deal with many adverse effects that natural disasters may bring, maintain social stability, and ensure the safety of citizens who are hindered by the management system, it is imperative to establish a complete set of a scientific emergency management system. The management system has formed a professional team in the management system of urban flood disaster, that is, focusing on public security and armed police and taking flood control professional team as the basic management system strength and emergency volunteers as the auxiliary force. At present management system, there are many management systems in the research of emergency rescue. Aiming at the discussion of rescue mechanism, framework, planning, and other aspects, an effective emergency rescue command system is the premise for the management system to effectively implement the emergency management system. The management system expounds on the process of emergency management of the emergency management system from the medical point of view: the first stage is the crisis-brewing stage, that is, the symptom period of the crisis, and the emergency management system with signs that shows the possibility of the crisis; the second stage is the outbreak stage of the crisis, that is, the occurrence period of the crisis. The crisis has been triggered by the emergency management system and may endanger the survival and development of society. The third stage is the diffusion stage of the crisis, that is, the crisis continues the emergency management system period, and it spreads after the crisis occurs, which is also a stage of eliminating the crisis; the fourth stage is the crisis management and emergency management system and recovery stage, that is, the crisis recovery stage, in which the crisis has been solved. Management system in the process of dealing with urban flood disaster, the most commonly used management system practice at present, is still to implement an emergency management system. However, the emergency management system needs experts to formulate management system according to domain knowledge and active judgment, which has high requirements for event domain knowledge, and the regulations of the management system are often general and abstract. The poor operability and feasibility of the actual management system have always been a relatively concerned and controversial issue.

The emergency management system has the function of emergency planning, program, and guide, is the carrier of emergency ideas, is the publicity management system book, mobilization order, and charge number of emergency actions, and is the key link for the government emergency management department to implement the management system of emergency education, prevention, guidance, and operation. Generally speaking, the natural disaster emergency management system mainly focuses on the construction of “one case, three systems.” The system structure is shown in Figure 2 below.

Management system in the county-level government shall, in light of the actual situation, conduct a systematic investigation of all kinds of hazard sources, factors, regional and social conflicts, and disputes in its jurisdiction, at the same time, establish a detailed database of hidden dangers' investigation, and carry out targeted monitoring and classified management of dynamic and emergency management system according to the local actual situation. In addition, the formulation or modification cycle of an emergency management system is relatively long. Usually, the formulation of an emergency management system will take several years to be modified and improved, which will cause the problem of whether the management system is suitable for the actual needs of the current social and economic background in the later period. Therefore, the monitoring and early warning system is composed of elements such as police identification, risk assessment, information early warning, and emergency management system. Each of the elements of the emergency management system has different functions, and together they form an interrelated organic whole. Only by establishing a scientific, effective, and well-functional management system can the management system link and organize all links in various accidents, so as to achieve the goal of reducing the disastrous consequences of the accident management system, ensuring personnel life safety, reducing property losses, and restoring and rebuilding as soon as possible.

The functions of the monitoring and early warning system of the management system include the following: the emergency management system shall do a good job in monitoring and prediction and prior risk assessment, predict the possibility of disasters and rapid response when disasters occur, and shall make emergency preparation, protect people and things, activate the positive response system, and reduce disaster losses. Management system to develop an emergency management system for natural disasters can reduce unreasonable behaviors in the management of natural disaster emergency management system and make the emergency management of natural disasters more scientific and reasonable. If the management system can be rectified in a short time, the hidden dangers shall be immediately eliminated; if the rectification is difficult and needs to be carried out for a long time, it is necessary to formulate a perfect rectification scheme of the emergency management system, complete it within a time limit, and do a good job in monitoring the emergency work; if it is difficult to complete the emergency management system, it shall timely report to the superior government. The emergency management system of a natural disaster management system is generally based on comprehensive disaster prevention planning. Its major subsystems mainly include the following: perfect self-management system, natural disaster emergency organization, management, and command system; strong natural disaster emergency engineering rescue guarantee system; the comprehensive management system, which is a mutual support system that coordinates and freely responds; a secure supply system for adequate disaster preparedness; and emergency rescue team reflecting the management system of comprehensive rescue.

## 4. Application Analysis of Scenario Construction Technology in Emergency Management

### 4.1. Scenario Construction Technology

Scenario construction is based on regional risk assessment and system vulnerability analysis to make scientific assumptions about the possible event scenarios with extremely serious consequences in a certain period of time in the future, build the evolution process under the general law of scenario events, simulate and calculate the accident consequences, and sort out the emergency task list to be taken to deal with scenario events. It is a technical method to evaluate the actual emergency capability against the target capability required to complete the task and put forward suggestions and measures to improve the emergency preparedness capability. More than 50 million hectares of crops were affected, more than 300 million people were affected, more than 4 million people were urgently relocated, thousands of people died, about 5 million houses collapsed, and there was a direct economic loss of more than 150 billion yuan. The comparison of disaster losses between 2020 and 2021 is shown in Figure 3 below.

“Scenario construction” is essentially a process of risk analysis and hazard identification, which makes scientific assumptions about possible and potential emergencies in a certain time in the future, and through the analysis and simulation of this hypothetical scenario. Its evolution process and consequences are reasonably inferred, and the tasks to be completed are summarized in order to deal with the situation, so as to identify the shortcomings of its own system. The research process of putting forward targeted prevention and emergency preparedness measures is generally composed of four levels, two guarantee systems, and four service objects. Suppose a secondary indicator *S*_*Bi*_ has K corresponding tertiary indicators *S*_*Ci*_, the scoring formula of the secondary indicator *S*_*Bi*_ is as follows:

(1) $$\begin{array}{c} S_{Bi}=\sum_{i=1}^{k}W_{3i}S_{ci}. \end{array}$$

Police situation identification pays more attention to the time, place, and nature of disasters, tracks disaster risk factors by using modern information technology, and transmits the collected information and data to managers; local governments should use advanced technical means to continuously track disaster risk factors to ensure the objectivity, accuracy, and comprehensiveness of data and information. The technical basis of “scenario construction” is as follows: three core elements: scenario, consequence, and task. There are four layers, including three-dimensional measurement and control platform of internet of things, information-sharing network, business support platform, and decision software platform; the two guarantee systems include mature and advanced technology system and coordinated and powerful policy system; the four service objects include water conservancy departments, municipal departments, competent leaders of municipal government, and social public users; the social public obtains information services by visiting the website. After calculating the similarity between the target case and the historical cases in the case candidate set, the historical cases with high similarity need to be extracted as suitable cases. In the subrule basis, the comparison of basic probability allocation values of different rules is shown in Figure 4 below.

Under the influence of the planned economic system, the disaster management system gradually formed in China is a single management mode by category and subsector under the unified leadership of the central government, that is, each disaster or several related disasters are, respectively, responsible by one or several related departments. The scoring method for emergency preparedness capability of situational events is as follows:

(2) $$\begin{array}{c} S=\sum_{i=1}^{4}W_{1i}S_{Ai}. \end{array}$$

Emergency preparedness is developed by “scenario construction”: diagnosis and evaluation of emergency preparedness ability; targeted suggestions on preparation ability are put forward; the emergency plan is improved. Emergency capability refers to the emergency capability required for each task according to the emergency task list and the description of the situation consequences and required response actions and lists various emergency capabilities for the situation response. The ability elements are evaluated item by item, and the evaluation results are shown in Figure 5.

There are some deficiencies in this vertical management. For example, the management of various disasters is independent of each other, there is a lack of unified overall coordination, and there are often repeated constructions among various disasters. Especially in the construction of basic geographic information, communication network, and disaster relief equipment and team, low-level reconstruction is quite common. This has affected the effectiveness and rationality of national investment in disaster reduction. The method of setting a similarity threshold in advance can be used to accurately extract suitable historical cases. Note that it indicates the similarity threshold between the target case and the historical case, and its calculation formula is as follows:

(3) $$\begin{array}{c} \xi =\rho \text{max}\left(\sin\left(Z^{*}\cdot Z_{l}\right)|l\right). \end{array}$$

Therefore, it is necessary to combine scenario construction technology with emergency preparedness capability evaluation, take the emergency tasks sorted out in the scenario construction process as the guidance, compare the target capabilities needed to complete the emergency tasks with the actual capabilities, analyze the capability gap of each emergency task, and comprehensively evaluate the emergency preparedness capability.

According to the analysis of rescue measures for specific events or tasks, due to the wide variety of accidents and disasters in cities, complex situations, strong emergencies, and large coverage, emergency activities involve all levels from senior management to grass-root personnel, from public security, medical treatment to environmental protection, transportation, and other fields, which have brought many difficulties to daily emergency management and emergency rescue command. Therefore, it is necessary to use scenario construction technology to mobilize and coordinate functional departments, establish a scientific and perfect emergency system, and implement standardized and orderly standardized operation procedures. Scenario construction is the realization and application of “bottom-line thinking” in the field of emergency management. “Prepare from the worst and strive for the best results.” The scenario events constructed by it are typical and represent the highest risk in the region.

### 4.2. Evaluation and Analysis of Emergency Preparedness

Emergency preparedness capability belongs to the category of capability. Its purpose is to reduce the occurrence probability of events/accidents, reduce casualties and property losses, and control the impact range of event/accident consequences. It covers the organizational system of emergency management, emergency plan, emergency command, emergency support, and other aspects. Its main influencing factors are human, material, financial, technology, and management. According to the scenario evolution process and combined with the characteristics of existing flood control emergency management, the emergency task analysis is divided into four stages: flood control preparation stage, monitoring and early warning stage, emergency response stage, and recovery and reconstruction stage. According to the scenario construction, the emergency response volume in four stages of drought river flood disaster emergency task is shown in Figure 6.

Emergency management refers to an organized, planned, and continuous dynamic management process, in which the government takes a series of control actions at different stages of crisis development in order to effectively prevent, deal with, and eliminate the crisis. The input information may be different in type and scope. According to the evaluation grade, there are qualitative or quantitative information transformation methods:

(4) $$\begin{array}{c} S\left(A^{*}\right)=\left\{\left(a_{ij},\gamma_{ij}\right);j=1,\ldots ,J_{i}\right\}. \end{array}$$

The emergency plan of the historical case with the greatest similarity with the target case obtained through case retrieval is not necessarily the optimal emergency plan, because, in the actual emergency disposal process, the decision-maker must consider whether the implementation effect of the emergency plan is satisfactory. Emergency linkage is a comprehensive innovation in concept, system, technology, and means based on the traditional treatment methods in the past. Assuming that the input value of the premise attribute is A^*∗*^, it can be converted into a confidence structure by the following formula:

(5) $$\begin{array}{c} S\left(A^{*}\right)=\left\{\left(A_{ij},\gamma_{ij}\right);j=1,\ldots ,J_{i}\right\}. \end{array}$$

The key points of emergency management are as follows: obtaining crisis information and early warning; crisis preparation and prevention; crisis control and response; postcrisis recovery and reconstruction; and continuous learning and innovation. Because the natural disaster crisis is very sudden and destructive, the environment in the area where the natural disaster crisis occurs is very complex, and the time left for rescue workers is also very limited. Therefore, natural disaster crisis management has a strong urgency, which requires the crisis managers to quickly and flexibly respond. The 24-hour duty system of county-level governments is established and improved, the smooth flow of information transmission channels is ensured, information submission commissioners are set up in key industries and regions, and the people to report relevant information to the county-level governments in time are encouraged. In combination with the characteristics of scenario events and the evaluation index system of emergency preparedness capability, and according to the opinions and suggestions of experts and staff in the chemical industry zone, in order to accurately reflect the impact of each level of indicators on the evaluation object, Figure 7 below is the analysis of emergency response indicators.

The early warning and release mechanism of flood disaster information is established and improved, and full use of various publicity media and communication networks such as radio, television, newspapers, and mobile phone text messages are made to release early warning information in time. In the trained confidence rule base system, after the input information is given by the expert, the activation rule weight is determined by combining the input information, rule weight, and premise attribute weight, and then, the activation weight of the confidence rule is calculated as follows:

(6) $$\begin{array}{c} \omega_{k}=\frac{\theta_{k}\prod_{i=1}^{M}\left(\gamma_{i}^{k}\right)}{\sum_{l=l}^{L}\theta_{l}\prod_{i=1}^{M}\left(\gamma_{i}^{k}\right)}. \end{array}$$

The channel of information dissemination is smooth, and we are committed to building an early warning information network with wide coverage. Because the emergency effect evaluation of urban flood cases involves many aspects, the evaluation grade is generally qualitative description, and there is some uncertainty, which is a multiattribute objective decision-making problem. Linkage mechanism is a comprehensive service system, which can mobilize the police forces of different departments and police districts in the shortest time to cooperate with each other and make an orderly, rapid, and efficient response to public emergencies.

The establishment of the emergency preparedness mechanism mainly includes three aspects: first, the organization system and operation mechanism of emergency management are established. Second, an early warning system is established. A scientific early warning system can prevent and reduce the possible losses caused by natural disasters to the greatest extent. Third, training and drills are established. The rehabilitation mechanism of natural disasters is the recovery and reconstruction mechanism of natural disaster emergency management. When a flood disaster occurs, the county government should quickly respond, carry out pretreatment, focus on rescuing the people in distress, and fully carry out rescue and disaster relief. At the same time, necessary measures should be taken to prevent secondary and derivative disasters. The recovery and reconstruction submechanism plays an important role in the mitigation, recession, and elimination of emergencies, mainly in order restoration, facility reconstruction, personnel resettlement, psychological rehabilitation, independent investigation, and organizational change.

## 5. Conclusions

A natural disaster is one of the most serious disasters in human society. It causes great damage, poses a great threat to towns and villages, and brings great harm to people's lives and property. The emergency management system of urban flood disaster based on scenario construction technology is an artificial intelligence technology that simulates the intuitive thinking mode of human beings. Compared with other expert systems, its obvious advantages are as follows: it is not limited by domain knowledge, the reasoning process is simple, and the reasoning result is operability and incremental learning. The core goal of “scenario construction” technology is to solve the problem of “what should we do now and how to better deal with it in the future” for specific or different scenarios. In this study, an emergency preparedness assessment method based on scenario construction technology is proposed. This method can objectively reflect the gap between the actual and target capabilities of emergency preparedness for scenario events, so as to propose suggestions and measures that meet the actual needs and enhance the regional emergency preparedness. Introducing scenario construction technology into the field of urban flood disaster emergency decision-making can not only solve the bottleneck problem of knowledge acquisition of emergency plan but also solve the problem of describing the “uncertainty” and “unknown” information at the beginning of the disaster through the confidence structure expression mechanism of attribute similarity between urban flood disaster cases so that the emergency plan of urban flood disaster can be quickly generated even if the emergency decision-making information is missing. There are many kinds of urban emergencies with high uncertainty, which makes the types and quantity of emergency resources have higher requirements, and its workload is huge. As the disaster-causing mode has changed and will continue to change, the performance of scenario evolution in disasters will become more obvious. [30].

## Figures and Tables

**Figure 1:** Contents of emergency cases of urban flood disaster.

**Figure 2:** Composition of natural disaster emergency management system.

**Figure 3:** Comparison of disaster losses between 2020 and 2021.

**Figure 4:** Basic probability distribution value.

**Figure 5:** Evaluation results.

**Figure 6:** Emergency response volume in four stages of emergency task.

**Figure 7:** Analysis of emergency response indicators.

## Data Availability

All the data are available in the paper.
